RETRACTED

# Visual Corneal Photomechanical Analysis Is Combined with the Pentacam Correlation Index for the Diagnosis of Cone Corneas at Different Stages of Progression

**DOI:** 10.1155/2022/4682901

**Published:** 2022-02-21

**Authors:** Qiong Cheng, Feng Zhang, Tixian Tian, Lan Wu, Linna Li, Meixia Chen, Ye Zhou

**Affiliations:** ^1^Department of Ophthalmology, Taikang Tongji (Wuhan) Hospital, Sixin Road North, Wuhan 430050, China; ^2^Key Laboratory of Metallurgical Equipment and Control Technology, Ministry of Education, Wuhan University of Science and Technology, Wuhan 430081, China; ^3^Hubei Key Laboratory of Mechanical Transmission and Manufacturing Engineering, Wuhan University of Science and Technology, Wuhan 430081, China; ^4^Precision Manufacturing Institute, Wuhan University of Science and Technology, Wuhan 430081, China

## Abstract

Cone-shaped corneas are blinding eye diseases characterised by dilated and thinning corneal tissue and forward conical protrusions, most often in adolescents. Early detection and intervention can prevent further dilatation of the cornea. The prevailing examination methods and techniques are not difficult to diagnose clinical cone corneas, but there are limitations in the diagnosis of early cone corneas (static cone corneas and subclinical cone corneas). In this study, we investigated the diagnostic value of the combination of these two instruments in the diagnosis of clinical cone corneas and subclinical cone corneas by performing the Pentacam and Corvis ST examinations in healthy eyes and dystrophic cone corneas. This study provides a theoretical basis for early cone cornea screening and diagnosis. The analysis revealed that only TP, SPA1, ARTh, and bIOP were normally distributed among all included parameters, and only bIOP was normally distributed with equal variance. TBI and CBI indices have a certain sensitivity and specificity for the diagnosis of subclinical cone corneas, with a strong diagnostic ability, and can be used for screening and early diagnosis of cone corneas.

## 1. Introduction

The eye is an important visual organ for detecting the outside world and perceiving our surroundings. 80% of the information we receive from the outside world are received through the human eye. The human eye has a very complex structure, of which the cornea, located at the very front of the eye, is composed of transparent tissue that not only protects the eye but also provides 70% of the refractive index of the eye [1] and is the main refractive medium of the human eye, which means that small changes in the morphology of the cornea can lead to significant changes in the optical properties of the whole eye. Corneal diseases such as cone keratoconus, dilatation [2], and keratoconus surgery [3] can all lead to significant changes in the optical properties of the cornea.

RETRACTED

The cornea is mainly composed of five layers: the epithelium, Bowman's layer, stroma, Descemet's membrane, and endothelium, of which the thickness of unevenly distributed collagen fibres and extracellular matrix between the fibrous laminae, making the cornea nonlinearly elastic and viscous [4], and it has complex photomechanical properties such as anisotropy [5]. The photomechanical properties of the cornea are important and valuable for the diagnosis and therapeutic evaluation of ophthalmic diseases, especially corneal diseases such as glaucoma, keratoconus [1], limbic degeneration [6], and iatrogenic keratectasia [7] after corneal refractive surgery, and for the maintenance of corneal morphology. In addition, the photomechanical properties of the cornea can affect the measurement of intracellular pressure [8]. Therefore, studying the photomechanical properties of the cornea is of great importance and clinical application.

Cone cornea is a common noninflammatory corneal disease that manifests itself as a forward protrusion in the centre of the cornea and is prone to high myopia, irregular astigmatism, and varying degrees of deterioration in vision. Once severe cone cornea occurs, it will be irreversible and patients will eventually have to undergo corneal transplantation. Cone corneas tend to occur in adolescence (15–25 years), with a general average incidence of 5 per 1,000. The cause and pathogenesis of primary cone keratoconus are unknown, while secondary cone keratoconus is mainly caused by refractive surgery. If the biomechanical properties of the patient's cornea can be accurately determined before surgery, screening for risk corneas such as early cone corneas or subclinical cone corneas, postoperative follow-up assessment and modelling of corneal biomechanical parameters, and the risk of refractive surgery complications can be effectively reduced, and a system of early cone corneal diagnosis theory and methods can also be established, as shown in Figure 1.

The diagnosis of preclinical cone corneas has always been a challenge for ophthalmologists because of the lack of obviousness of early cone corneas on topography and clinical signs as well as the overlap and low sensitivity of clinically specific indicators between subclinical cone corneas and some morphologically abnormal or thin normal corneas. Although there are many new devices and new parameters or indices for the diagnosis of early cone corneas, new cone grading systems have been reported in the literature. There are still deficiencies in the diagnosis of early cone corneas.

RETRACTED

The TBI is an index calculated from tomography and photomechanical parameters based on an artificial intelligence method, i.e., the index contains both morphological and biochemical parameters of the cornea. In this study, comparing 15 indices and parameters in the normal group with the subclinical cone group, the index with the highest diagnostic power was the TBI, with an AUC of 0.980, a sensitivity of 96.00%, and a specificity of 98.88%. This indicates that this index is able to discriminate better between normal eyes and subclinical stage cone corneas than either tomography or the photomechanical index CBI, which is more sensitive. However, when comparing the normal group of the trophoblastic cone group, the sensitivity of the TBI was only 67.65%. The specificity was 75.28%, and the AUC was 0.774. This indicates that the TBI index has some reference value for clinicians to screen for cone corneas. However, it has low sensitivity and specificity in distinguishing normal corneas from trophoblastic cone corneas and is used to screen patients with trophoblastic cone corneas with low diagnostic ability. Sergienko and Shargorodska [9] found no significant correlation between TBI and K values in conical corneas compared to normal patients. Also, Bae et al. [5] showed that TBI did not correlate significantly with IOP and corneal thickness as well, which are precisely the two factors that have the greatest impact on corneal biomechanics. Therefore, TBI can be a more reliable indicator for the diagnosis of early cone corneas than CBI.

It has been shown that although early cone corneal topography is not abnormal, changes in the viscoelasticity of the cornea due to changes in the internal structure of the cornea have led to changes in the biomechanics of the cornea itself, which are directly or indirectly related to the collagen synthesis of the cornea [10], meaning that cone corneas do not initially have morphological abnormalities in the earliest stages but generally have photomechanical abnormalities. Biomechanical changes often precede changes in corneal topography. Guo et al. [11] concluded that cone corneas do not have morphological abnormalities at the beginning but generally have photomechanical abnormalities. In this study, to assess the ability of corneal biomechanics in the diagnosis of early cone corneas, some important parameters of Pentacam and Corvis ST were included simultaneously. The sensitivity of the CBI index was 80.00%, and the specificity was 98.88%, when comparing the 15 indices and parameters in normal and subclinical cone corneas. It has a high diagnostic power. The sensitivity of the CBI was 82.35%, and the specificity was 38.20%, with an AUC of 0.621. This indicates that the CBI index is a useful reference for clinicians in screening for cone corneas. It has a higher sensitivity than that of the TBI index in distinguishing normal corneas from static cone corneas but a significantly lower specificity than that of the TBI index and has a lower diagnostic ability for screening patients with strong cone corneas. Zhang et al. [12] found that the CBI index AUC area and specificity were less than those of the TBI in the diagnosis of subclinical cone corneas, which are consistent with the results of this study, as shown in Figure 2.

RETRACTED

This study evaluated the diagnostic ability of modern medicine for cone corneas at different stages of progression and provided some reference for the diagnosis of early cone corneas in clinical work, but there are still some shortcomings; for example, this study did not conduct further grading analysis to compare the severity of cone corneas in the clinical stage, the difference in the inclusion criteria of the group of cone corneas, and the limitation of the sample size will affect the results of this study, so the results of this study still need to be validated by a larger sample size.

## 2. Related Work

Current clinical methods for the diagnosis of corneal diseases (e.g., conical cornea) are mainly based on corneal morphological features, such as corneal topography [13], Pentacam anterior segment analyzer, optical coherence tomography (OCT), and ultrasound biomicroscopy (UBM) [7]. However, corneal morphology can only be diagnosed with the help of ultrasound biomicroscopy (UBM) [14]. However, corneal morphological methods can only capture static features of the human eye and are susceptible to ocular surface diseases and tear film, and for some cone corneas, morphological changes are later than structural intensity changes [7], especially since some cone corneas have similar morphology to normal corneas and cannot be screened by static corneal morphological analysis. This makes in vivo measurements of photomechanical properties of the corneal tissue such as elasticity and viscoelasticity particularly important. The lack of a comprehensive in vivo corneal photomechanical measurement technique in clinical practice poses a significant risk and uncertainty of corneal refractive surgery.

Corvus ST is a noncontact dynamic corneal visualisation technique combining the Scheimpflug ultra-high-speed camera and impulse pressure technology to provide a real-time dynamic recording of the entire process of corneal compression deformation and deformation reduction, providing important mechanical parameters with good repeatability and consistency.

RETRACTED

In recent years, corneal photomechanical parameters have been a hot topic of research. For example, some studies have analysed the prediction of corneal photomechanical parameters by numerical simulation [15] and the measurement of intracellular pressure [16]. Some studies have been devoted to corneal hysteresis and its association with glaucoma [17], thickness measurements, or hysteresis measurements in children and healthy subjects, studying the relationship between the cone cornea and its photomechanical properties. The establishment of corneal photomechanical measurements by different ophthalmometers to measure corneal photomechanical properties in various ophthalmic diseases has become a research hotspot in the field of ophthalmology or corneal biomechanics, with an urgent clinical need and research value.

Vlasák et al. [18] proposed some new parameters such as the corneal indentation area (D_area_), corneal contour deformation (CCD), corneal creep rate (V_creep_), energy absorbed area (A_absorbed_), and tangent stiffness coefficient (STSC) [19]. Elkitkat et al. [20] found that all parameters of Corvis ST output were significantly different between the cone and normal corneal groups. Fares et al. [13] found that four parameters 1AL, 2AL, HC radius, and deflection length at the highest concavity were significantly different between cone and normal corneas. Tekin et al. [21] found that all parameters of Corvis ST output were significantly different between cone and normal corneas. Li et al. [22] found that all parameters of Corvis ST output were significantly different between cone and normal corneas. found that all parameters of Corvis ST output were significantly different between cone and normal corneas. The Corvis ST was used to compare the biomechanical properties of the cornea between dry and healthy eyes. Yi et al. [23] found that the parameters extracted from the Corvis ST were used to differentiate between normal and cone corneas by combining the different properties of the parameters extracted from the Corvis ST.

## 3. Corvis ST-Based Corneal Biomechanical Testing

Corvis ST is a noncontact, dynamic visualisation technique for quantitative and qualitative analysis of corneal biomechanical properties, which is rapidly gaining interest in the field of ophthalmology and other fields due to its rapid measurement, noncontact, automated acquisition, and “open” dynamic visualisation of parameters throughout. The air pressure is measured three times in succession by an analogue acquisition card (model NI-USB6211) with a sampling rate of 50 Hz. The air pulse is sprayed onto the hemispherical apical surface, and the air pressure equation is

(1) $$\begin{array}{c} P_{air\;}=P\left(r,t\right), \end{array}$$

where *r* denotes the radius of the air pressure, the shape of the air pressure obeys a Gaussian distribution, and *t* denotes time. The air pressure measured by the pressure sensor is calculated as follows:

(2) $$\begin{array}{c} f\left(t\right)=\int_{0}^{2\pi }\int_{0}^{2\pi }\left[P\left(r,t\right)\cos\;\theta \right]\left(R\;d\theta \right)\left(R\;\sin\;\theta \;d\theta \right)\\ =2\pi R^{2}\int_{0}^{2\sigma }P\left(R\;\sin\;\theta \;d\theta \;,t\right)\sin\;\theta \;\cos\;\theta \;d\theta \text{.} \end{array}$$

After integration, the air pressure as shown in Figure 3, *f(t)* can be represented by the Gaussian model:

(3) $$\begin{array}{c} f\left(t\right)=a_{1}\cdot e^{-{\left(\frac{t-b_{1}}{c_{1}}\right)}^{2}}+a_{2}\cdot e^{-{\left(\frac{t-b_{2}}{c_{2}}\right)}^{2}}\text{,} \end{array}$$

where *a*_1_, *a*_2_, *b*_1_, *b*_2_, c_1_,  and c_2_ are the model coefficients [10].

RETRACTED

## 4. Case Studies

### 4.1. Information

Patients and volunteers who attended our hospital from November 2017 to November 2019 with a confirmed diagnosis of conical cornea were included in the study. A total of 154 subjects were included in this study, of which 65 patients with conical corneas were classified as clinical: 44 eyes, subclinical: 50 eyes, and strong: 34 eyes. There were 89 normal volunteers, 89 eyes. The mean age of the cone group was 36.37 ± 10.13 years, of which 44 eyes were in the clinical phase, accounting for 34.37% of the cone patients; 50 eyes were in the subclinical phase, accounting for 39.06% of all cone patients; and 34 eyes were in the thrombolysis phase, accounting for 26.56% of the cone patients. Patients with advanced cone corneas were excluded due to extreme abnormalities in the morphology and the unreliable quality of the values generated by multiple measurements. Patients and volunteers undergo myopic laser surgery (normal group): 89 patients, 89 eyes.

All patients underwent a comprehensive ophthalmic examination, including patient's distance visual acuity, slit-lamp examination, noncontact IOP examination, computerised optometry and corrected visual acuity, triple-lens examination, and Pentacam and Corvis ST examinations of acceptable quality. All patients stopped wearing soft contact lenses for at least 1 week and hard contact lenses for at least 3 weeks prior to the examination, and all patients did not use any eye drops other than artificial tears. Both the Pentacam and Corvis ST examinations were performed by the same experienced medical technician.

Anser and Mcmahon classified cone corneas according to their progression into stroke-stage cone corneas, subclinical cone corneas, and clinical cone corneas. The inclusion criteria for the normal group were as follows: no ophthalmic disease other than astigmatism and myopia, one eye selected at random, normal corneal topography in both eyes, and corrected visual acuity of 1.0 or more.

RETRACTED

The criteria for inclusion of cone-shaped corneas in the thrombolysis stage are as follows: refractive error only, no other symptoms or signs, and normal slit-lamp and corneal topography. Patients with cone corneas in the stroboscopic phase were included in the study if the eye had been diagnosed with clinical or subclinical cone corneas in the better eye, and the corneal topography of the better eye was not abnormal (maximum refractive error on the anterior surface of the cornea ≤46.5 D), best-corrected visual acuity ≥0.8, and no signs of cone corneas on slit-lamp examination.

The inclusion criteria for the subclinical cone angle group are as follows: history of refractive error in the affected eye, no other symptoms or signs, no significant abnormalities on slit-lamp examination, best-corrected visual acuity ≥0.8, and cone angle on corneal topography (central refraction >47D on the anterior surface of the cornea; the difference in refraction between the central 3 mm and lower 3 mm of the cornea >1.26D; and the difference in refraction between the central anterior surface of the cornea in both eyes >0.92 D).

The inclusion criteria for the clinical cone group are as follows: history of refractive error, best-corrected visual acuity <1.0, and typical corneal topographic changes in cone corneas with at least one of the following signs: Fleischer ring, Vogt's stripe, corneal stroll thinning, apical corneal scar, anterior corneal bulge, etc. Patients who met the diagnostic criteria for a clinical stage cone cornea in both eyes were included in this study group.

The abovementioned inclusion criteria for the cone cornea subgroup were based on the Rabinowitz diagnostic criteria and were in accordance with the 2015 Global Consensus on Cone Cornea Diagnosis.

### 4.2. Results

The most powerful parameter was BAD-D with a sensitivity of 64.71%, specificity of 84.27%, AUC of 0.781, 95% confidence interval of 69.8% to 85.1%, *Z* = 5.650, and *p* < 0.001, followed by TBI with a sensitivity of 67.65%, specificity of 75.28%, and AUC of 0.8063. This was followed by TBI with a sensitivity of 67.65%, specificity of 75.28%, AUC of 0.774, 95% confidence interval of 65.2% to 81.5%, *Z* = 4.639, *p* < 0.001, and Youden index of 0.4293. Although all parameters or indices except DA ratio (*p*=0.0787) and bIOP (*p*=0.1296) had *p* values less than 0.05 for the ROC curve, indicating that all parameters or indices except DA ratio and bIOP had the ability to predict cone corneas in the clinical phase of the trophoblastic period. According to nonparametric tests, bIOP, CBI, Df, Db ARTh, integrated radius, DA ratio, and SPA1 were not statistically significantly different (*p* > 0.05), so none of the abovementioned parameters or indices was statistically significant in the diagnosis of thrombolysis cone corneas. Therefore, only BAD-D, TBI, Da, Dt, Dp, Kmax, and TP have some predictive diagnostic ability in the diagnosis of stuttering cone corneas, but the diagnostic ability is poor. See Table 1 and Figures 4 and 5 for details.

RETRACTED

In the normal group and the subclinical cone group, the first 6 parameters or indices of the ROC curve area were BAD-D, TBI, Dp, Kmax, Dt, and integrated radius, and the *p* value of the ROC curve was greater than 0.05. Therefore, there was no significant difference between the abovementioned 6 parameters or indices in the diagnosis of the subclinical cone cornea. In the normal group, the first 6 parameters or indices were TBI, BAD-D, Dt, Da, ARTh, and CBI compared with those of the subclinical conical cornea group, of which the three major indices TBI, BAD-D, and CBI were not statistically different from each other in terms of ROC surface area (*p*=0.667). TBI was statistically different from CBI (*p* < 0.005). There was no statistical difference between BAD-D and CBI (*p*=0.109). When comparing normal versus clinical stage cone corneas, the top 6 parameters or indices of diagnostic ability were TBI, BAD-D, Da, TP, CBI, and Kmax, all of which had a *p* value greater than 0.05 between them, and none of these parameters or indices were statistically different in the diagnosis of clinical stage cone corneas. For details, see Table 2, and Figures 6 and 7.

## 5. Corvis ST-Based Corneal Biomechanics In Vivo Procedure

In this experiment, all subjects underwent a complete ophthalmologic examination. All measurements are performed by two specialist ophthalmologists, who diagnose whether the cornea is conical or not. Measurements were made with a shear reflex on the retina or a steep central or near paracentral reflex on funduscopic examination and corneal topography, and the diagnosis of a conical cornea was made using at least one of the following slit-lamp signs: Vogt stripes, a Fleischer ring greater than 2 mm in diameter, or a corneal scar that is consistent with a conical cornea, as shown in Figure 8.

During the Corvis ST measurement, the subject, in conjunction with an eye care professional, places the lower jaw on the mandibular rest and the forehead on top of the frontal rest, adjusting the position of the mandibular rest so that the subject blinks and then looks at the red dot with both eyes fixed on the target. The pressure head is aligned with the cornea and automatically identifies the cornea and applies air pressure evenly to the cornea, causing the cornea to deform under pressure and gradually reverting the deformation as the pressure decreases. As shown in Figure 9, the Corvis ST uses the Scheimpflug high-speed camera to record corneal deformation at a frame rate of 4330 frames per second, with an acquisition time of approximately 30 ms. 139 frames of video are recorded per cornea, scanned at 8.5 mm horizontally, with an image resolution size of 200 ∗ 576 pixels, converted to physical size at a rate of 0.0156 mm/pixel horizontally and 0.0165 mm/pixel vertically.

RETRACTED

In this dataset, there are 175 corneal data of subjects, including 100 normal corneas and 75 keratoconus. Among the subjects with keratoconus, if only one eye is diagnosed as keratoconus, that eye was selected for measurement. If both eyes are diagnosed as keratoconus, one was selected at random for measurement [24]. The subjects did not have corneal or eye surgery, nor did they have any eye diseases other than keratoconus or any other diseases affecting the eyes. The data were collected in Tianjin Eye Hospital, Beijing PLA General Hospital, and Beijing Tongren Hospital. All subjects signed informed consent in accordance with the “Declaration of Helsinki.” The subject information table is shown in Table 3.

Therefore, in this experiment, 100 videos of normal corneas and 75 videos of conical corneas were acquired based on the Scheimpflug high-speed camera, each containing 139 frames of image sequences, for a total of 34,325 corneal images. Figure 9 shows the schematic diagram of the Corvis ST acquisition data, and the results obtained are shown in Figure 10.

As shown in Figure 10, the Corvis ST system provides the intracellular pressure and some photomechanical parameters based on the image analysis of corneal pressure deformation. However, in practice, artefacts such as tears, eyelashes, and other impurities often occur during acquisition, making the image analysis algorithm of the Corvis ST system perform poorly, seriously affecting the accuracy of the parameters calculated by the Corvis ST system.

## 6. Conclusions

In this study, the diagnostic value of the combination of these two instruments in the diagnosis of subclinical and clinical cone corneas was investigated by performing the Pentacam and Corvis ST examinations on healthy eyes, thrombolysis cone corneas, subclinical eyes, and clinical cone corneas and by statistically analysing 15 parameters or indices of the two devices. The test group was divided into three groups, namely, the subclinical cone group, clinical core group, and strong group. The analysis revealed that only TP, SPA1, ARTh, and bIOP were normally distributed among all included parameters, and only bIOP was normally distributed with a chi-squared.

RETRACTED

## Figures and Tables

**Figure 1:** Structure of corneal components.

**Figure 2:** Schematic diagram of the morphology of the orthokeratology and conical cornea.

**Figure 3:** Jet pressure variation curve with time.

**Figure 4:** Comparison of the six anterior cone corneal parameters AUC in the normal group with those in the stentorian phase.

**Figure 5:** Comparison of the AUC of the six anterior cone corneal parameters between the normal and subclinical group.

**Figure 6:** Comparison of the six anterior parameters of the AUC between the normal and conical corneas.

**Figure 7:** Comparison of AUC of parameters CBI, TBI, and BAD-D.

**Figure 8:** View from different perspectives.

**Figure 9:** Different observation effects.

**Figure 10:** Image taken by the Scheimpflug high-speed camera during the air-pressing of the cornea.

**Table 1:** Two-by-two comparison between groups.

Parameter	Normal group vs frustrated group	Normal group vs subclinical group	Normal group vs clinical group	Subclinical group	Frustration stage group vs clinical stage group	Subclinical group vs clinical stage group
TP (mm)	<0.01	<0.01	<0.01	<0.01	<0.01	0.032
BAD-D	0.014	<0.01	<0.01	<0.01	<0.01	0.094
Df	0.193	<0.01	<0.01	<0.01	<0.01	0.030
Db	1	<0.01	<0.01	<0.01	<0.01	0.036
Dp	0.007	<0.01	<0.01	<0.01	<0.01	0.068
Dt	0.017	<0.01	<0.01	0.013	<0.01	0.133
Da	0.006	<0.01	<0.01	<0.01	<0.01	0.043
Kmax (D)	0.002	<0.01	<0.01	0.021	<0.01	0.002
ARTh	1	<0.01	<0.01	<0.01	<0.01	0.02
CBI	0.023	<0.01	<0.01	<0.01	<0.01	0.11
TBI	0.035	<0.01	<0.01	<0.01	<0.01	1
Integrated radius	0.832	<0.01	<0.01	<0.01	<0.01	1
DA ratio	0.184	<0.01	<0.01	<0.01	<0.01	0.053
bIOP (mmHg)	0.174	0.359	0.029	0.002	<0.01	0.032
SPA1	0.65	<0.01	<0.01	<0.01	<0.01	0.015

**Table 2:** Means or medians for each parameter in the different progressive cone cornea groups.

Parameter	Median			
	Normal group	Setback group	Subclinical group	Clinical stage group
Df	0.11	0.78	3.34	11.09
Db	0	0.28	3.10	10.03
Dp	1.09	2	4.24	8.7
Dt	−0.07	0.65	2.23	3.02
Da	0.92	1.77	0.39	3.14
BAD-D	1.25	1.77	3.91	9.75
CBI	0.01	0.06	0.87	1
TBI	0.23	0.36	1	1
Kmax	44.2	45.25	47.9	46.65
Integrated radius	7.6	8.5	9.5	10.6
DA ratio	4.2	4.3	7.8	5.4

**Table 3:** Subject information (gender, age, and intraocular pressure).

	Normal group (*n* = 100)	Keratoconus group (*n* = 75)
Gender (male/female)	62/38	42/33
Age (years)	27.88 ± 6.55	24.72 ± 5.23
Intraocular pressure (mmHg)	14.01 ± 2.27	13.72 ± 2.71

RETRACTED

## Data Availability

The datasets used during the current study are available from the corresponding author on reasonable request.
